The article "A Region-Based Statistical Shape Modeling on the First Trapezoid-Metacarpal" was published in 2023. Journal: Appl Bionics Biomech.

# A Region-Based Statistical Shape Modeling on the First Trapezoid-Metacarpal

**DOI:** 10.1155/2023/3257460

**Published:** 2023-02-01

**Authors:** Lin Fu, Kaczmarek Łukasz, Ci Jiang, Yaodong Gu

**Affiliations:** ^1^Faculty of Sports Science, Ningbo University, Ningbo, China; ^2^Institute of Materials Science and Engineering, Lodz University of Technology, Lodz, Poland

## Abstract

A statistical shape model (SSM) based analysis was conducted in our study. We indicated the morphological differences of the first trapezoid-metacarpal (TMC) bone between the region-based statistical shape model (rSSM) and the nonregion-based statistical shape model (nrSSM). We aimed to characterize more specific and accurate variation results to detect and prevent osteoarthritis in an early way. CT image data of TMC from 31 healthy volunteers were simulated with 3D models. A training set of models was analyzed with principal component analysis, with both then- rSSM and rSSM. The region was identified automatically with Gaussian curvature analysis. We found four dominant shape variations from both nrSSM and rSSM. The rSSM showed more variations with fewer components compared with nrSSM. The first principal component revealed the size variation as the biggest component. A significant difference was presented in the second and the fourth principal component from rSSM, showing the torsion of the distal head of the first metacarpal which may increase the risk of osteoarthritis.

## 1. Introduction

Hand injury is going to be a major clinical problem for people, especially hand osteoarthritis (OA). It was reported that around 67% of women and 55% of men have such problem with their hands, which usually happens in the first trapezoid-metacarpal (TMC) joint, contributing to much possibility of pain of their hand OA [1]. However, what leads to the highest risk of TMC OA? The increasing number of mobile phone users and phone subscribers worldwide will be counted in. There are more than 2.4 million phone subscribers with 74% of all phone users texting messages worldwide [2]. Besides, as we know, with the rapid development of technology, the increasing request from communication and entertainment, have become indispensable in our daily life [3]. As prior studies hypothesized, biomechanical factors were considered, such as stress, strain, contact area, contact angle, and progression [4–6].

Anatomical feature of TMC could also be seen as another major factor relating to hand OA. According to the previous studies, finite element modeling (FEM) methods were mainly applied for implant design in most cases of surgery and clinical diagnosis. Based on computed tomography, analyzing TMC shape parameters could be essential for investigating the mechanism of osteoarthritis. Statistical shape models (SSMs) are a necessary way to quantify the variation of shape and classify morphological variation by decomposing shapes into a set of statistically significant modes (commonly principal components) [7, 8], based on the process of target image collection, modeling reconstruction, registering, and alignment. Rusli and Kedgley [9] used the SSMs for investigating the TMC shape variations, especially for the first two components, which could be necessary to find the most anatomical shape variations. In previous studies, there were processes of modeling reconstruction, finite element modeling, pathology classification, and prediction [8]. Furthermore, SSMs also allow us to investigate more about specific anatomical regions and find the significant location changes, which could be a major correlation to some hand injuries, such as ligament or internal diseases. Due to the limitation of measuring the torsion angle of 2D image, it is essential to measure and analyze it using 3D models with SSMs method. This shape analysis method allows to observe the widths, lengths, and tilt angles of TMC in a visible way, avoiding the difficulty and inaccuracy of 2D measuring [10, 11]. Region-based SSMs (rSSMs) analysis has been mentioned in earlier studies, for example, Zhang et al. [8] used the rSSMs in human femoral analysis, they compared the femoral shape variations with rSSMs and nonregional SSMs (nrSSMs), and they found that rSSMs showed more efficient location changes compared with normal SSMs. However, there were no studies making a comparison between rSSMs and the nonregional model using SSMs on TMC joint. In previous studies, regions were manually defined by drawing boundaries [12], which showed the limitation of accuracy, and more recent studies have used curvature as a metric for guiding or automatically defining region boundaries [13]. In our article, we classified the anatomic region using Gaussian curvature analysis. This method is applied in many areas, for instance, the 3D face detection [14], surface triangulation [15], and regional principal component analysis (PCA) [8].

There were other anatomical parameters of TMC joint, which have been observed in previous articles. Kim et al. [16] reported that articular tilt angles may have necessary effects on TMC disease, which could be an important factor leading to osteoarthritis [17, 18]. Usually, the normal nrSSM can measure the variation number and estimate the morphology factors on the subject, but rSSM not only can do the same measurement, but with much more precise analysis, it can indicate more accurate location and shape deformation on the subject. In this way, rSSM could be a beneficial way to make prevention from the diseases.

The purpose of this study was to investigate the differences between the rSSMs and nrSSMs on anatomic shape variations. But also by measuring five anatomical parameters, we hypothesized that anatomic features could be analyzed with accurate and correspondent rSSMs. Besides, rSSMs could quantify the regions independently with shape variations.

## 2. Materials and Methods

CT image data of TMC were obtained for the dominant hands from 31 healthy volunteers, consisting of 23 males (age: 46.86 ± 12.58 years) and 8 females (age: 39.60 ± 15.56 years). When the power was set at 0.8, the minimal sample size was obtained at 30. A SSM process was conducted to analyze the weights of principal components difference between rSSM and nrSSM, based on PCA.

### 2.1. Participant Information

All participants were volunteered to our study, and they were recruited to scan their wrists and thumbs in a clinically neutral position. All of them were using the right hand as their dominant hands. This study was approved by the Ethics Committee of the Faculty of Sports Science in Ningbo University, and all participants were informed about the study content.

### 2.2. Imaging

Each participant was asked to scan the hand in clinically neutral position with scanner parameter setting of 80 kvp and 80 mA, slice thickness of 0.625 mm, in-plane resolution of 0.4 mm × 0.4 mm, and pixel size of 0.488. The first trapezoid-metacarpal joints were segmented using Mimics v12.11 (Materialise, Leuven, Belgium) and 3D bone models were exported as meshed surfaces with 3-Matic Research 13.0 (Materialise, Leuven, Belgium). All CT raw scans were introduced to the software of Mimics, the bones were generated and simulated as 3D modelings. Exporting the 3D modelings to the software of 3-Matic research to operate smoothing and meshing, the best size of grids and high quality of meshing of the bones were obtained. The vertices of these surfaces were extracted to produce a training set of point clouds for SSMs generation.

### 2.3. Statistical Shape Model

Statistical shape model was implemented with a training set. Basically, nrSSM method consisted of serial processes (Figure 1). The first process was to simulate 2D images to 3D model in software Mimics. Then we checked the surface quality, choosing the lowest root mean square of 0.15 mm as a template target for preparing, registering, and aligning with the rest TMC models. After fitted meshes, TMC models have been registered as individually. The last step was to align all 3D models with target model. Registration and alignment were implemented using rigid coherent point drift [19]. PCA was carried out after model alignments, this process aimed to obtain a shape model. A final PCA was performed on the nodal coordinates of the training set meshes to yield the statistical shape model. Usually, the target limited number of principal components should be set at *n* − 1, where *n* is the total number of 3D samples of study database [20].

#### 2.3.1. Region-Based Statistic Shape Modelling

In our study, we divided rSSM into two steps, including the clustering step and the SSM training step [8]. In the clustering step, we collected all 3D models for automatically selecting the similar regional curves using Gaussian curvature analysis, according to the surface feature of concave and convex, showing the positive and negative curve analysis values. Finally, the most correspondent and correlative morphology regions were identified across the training set (Figure 2(a)). During the step of rSSM training, PCA was conducted on the regional 3D samples after clustering, involving processes of fitting, registering, and alignments. According to the previous study, Kim et al. [21] used tensor voting theory to classify the vertices; however, in most experiments, Gaussian curvature can show us automatically the region identified [8].  Figure 2(b) shows the definition of the anatomical locations of the first metacarpal bone.

#### 2.3.2. Principal Component Analysis

PCA was used in many studies. This method aimed to reduce the dimension, determining the most effects on morphological variations in this study [22]. Especially, the limited number of principal components was *n* − 1, where *n* is the sum number of subjects [20]. Target 3D bone model template was chosen as a reference object, other 3D bone models were used to conduct the registration and alignment, following the Generalized Procrustes analysis [23]. The distance between principal components shape model and mean shape model was calculated with cloud compare (http://www.danielgm.net/cc/).

(1) $$\begin{array}{c} x=\bar{x}+\sum_{i=0}^{n}w_{i}\Phi_{i}. \end{array}$$

In our study, *x* was defined as any shape variances in our training set, $\bar{x}$ was the mean shape obtained from the principal components *Φ*. The number of principal *n* was set as 6, where the accumulative variances were more than 80%. Thus, briefly, six weights were obtained from PCA, which need to be statistically analyzed in our study.

## 3. Results

As shown in Figure 3, total number of principal components was set as 10, and six principal components represented more than 80% of the total shape variances in our study. Both nrSSM and rSSM showed similar trends of the cumulative variation representation. The first and second principal components of nrSSM are 34.24% and 16.4%, respectively. Additionally, the first and second principal components of rSSM are 30.16% and 14.53%, respectively. There is a significant difference in PC1 between nrSSM and rSSM, but the difference was decreasing when more components were used. And for the first six components, the difference of cumulative variations of nrSSM and SSMs was increased. The rSSM explained more variations using less components than nrSSM.

Figure 5 shows the first four principal components of the first metacarpal bone with nrSSM, indicating the morphological variations in the first metacarpal bone. In the first principal component, a size variation was observed in the whole bone, especially at proximal and distal parts of the shaft. The second principal component shows a width difference at the anterior volar, especially at the proximal end of the shaft, as well as variation of thickness difference (Figure 4, PC2). Width difference can be also observed in the proximal end of shaft, according to the third principal component, plus the thickness difference can be seen at the medial part of shaft (Figure 4, PC3). An increased angle at the distal head can be found in the fourth principal component (Figure 4, PC4), and the flexion and extension of shaft can be also found (Figure 5, PC4).

As shown in Figure 6, the Gaussian curvature analysis results show that the value of rSSM was higher than nrSSM with −2SD model in all four principal components, as well as +2SD model. And the PC1 shows the highest Gaussian curvature value, following PC2, PC3, and PC4 with −2SD model and +2SD model for both rSSM and nrSSM, except PC4 with +2SD model. In +2SD model, significant differences can be seen at PC2 and PC4. The value of rSSM (0.51) was twice more than nrSSM (0.25). Besides, the significant difference can also be observed at PC4 with +2SD model, the rSSM (0.13) showed higher value than the nrSSM (0.32).

## 4. Discussion

The purpose of this study was to investigate the variation differences between region-based model and nonregion-based model using statistical analysis methods. We collected 31 healthy trapezoid-metacarpal joints' images in our study, performing a principal component weight analysis using nrSSM and rSSM on the first metacarpal bone. We hypothesized that it could be calculated independently when we used the nrSSM and anatomical features could be identified more precisely using region-based model, compared with nrSSM. We found that more and independent variation parameters could be found with nrSSM after Gaussian curvature analysis, confirming our first analysis. And there were significant differences indicating more and specific morphological variations that can be seen with nrSSM, compared with rSSM, confirming our second hypothesis.

Previous studies used the statistical shape models indicating the morphological variations in bones, including the human femur, knee, and trapezoid-metacarpal bones [8, 9, 24]. Lynch found that the first seven principal components of the SSM contributed more than 90% of shape variations between osteoarthritis and healthy knee, and the first principal component attributed to shape and size. In our study, the first principal component values were 30.16% (nrSSM) and 34.24% (rSSM), respectively, as shown in Figure 3. Combining the variation changes from −2SD to +2SD models in Figure 5, we can also find the size of the first metacarpal to become the most dominant variation. Schneider et al. [25] conducted a study to characterize size and shape differences between size-normalized shape model and nonsize-normalized shape model. They found that in the first principal component, the key variation is the size, not the shape, which was correlative to the result of our study (Figure 5, PC1).

According to the PC4 of +2SD model in Figure 6, a significant difference in Gaussian curvature value was presented between nrSSM and rSSM. Rusli and Kedgley [9] researched on the trapezoid-metacarpal bone, using SSM, to determine the correlation between the variability in anatomical features of the first metacarpal and trapezium. They defined the bending angle to calculate the relation between the shape of the bone and the shear force at the articular surface of the first metacarpal bone. In our study, there was a significant shaft bending and extension on the first metacarpal bone when using the rSSM. Increasing the bending angle leads to more shear force, which may weaken the ligament surrounding the joint [18]. In our study, PC4 showed the shape deformation in the sagittal plane, in both −2SD and +2SD models, the rSSM showed more precise results compared with nrSSM (Figures 3 and 6).

In our study, there was an obvious torsion angle at the first metacarpal bone in Figure 5 of PC2. As we know, the orientation of the first metacarpal bone is very important for the first trapezoid-metacarpal joint during daily functional motions. Increasing the torsion angle of the first metacarpal may cause higher risks of osteoarthritis [17]. In Figure 5 of PC3, there was a width difference at the distal and proximal head. Besides, Ladd et al. [10] found that the width of the trapezoid bone also could be a risk to cause osteoarthritis, the wider the facet, the higher the risk of osteoarthritis. The anatomical variations of the first metacarpal bone may have big influence on the performance of daily activities. We may need further research to figure out the associations between the morphology and kinematics of the first metacarpal bone.

In the previous studies, Zhang et al. [8] tried to use the rSSM on human femurs; they generated the regions automatically using Gaussian curvature analysis. Six anatomic regions were identified in this article; compared with nrSSM, the rSSM explained more variations using fewer components. We also got a similar conclusion in our study; less cumulative variation representing attributed to more variations can be found with nrSSM as shown in Figure 3. Gaussian curvature analysis is defining to characterize using normal vector voting. It was a necessary measurement for dividing the regions individually [26–28]. The individual regions are reliable and stable, which could be significant to get more accurate results.

It is also very important to mention the limitations of our study. We only divided the surface region into two individual parts; however, in the research of Zhang et al. [8], they defined six regions to make a comparison between nrSSM and rSSM, which may cause the result to be more reliable and accurate. The second limitation is we only tried this method on the first metacarpal bone, not on trapezoid bone also. In future research, we will continue to analye the whole trapezoid-metacarpal bone, plus observe the biomechanics features of this joint when conducting daily movements. The third limitation of this article would be the cartilage shape influences. In future, more specific research work will be conducted on the correlation between cartilage morphological variations and OA.

## 5. Conclusion

We applied SSM with two models, nrSSM and rSSM, respectively. Gaussian curvature analysis was used to divide the regions individually. Compared with nrSSM, rSSM not only showed more reliable and precise results, but presented more anatomic variations. To sum up, rSSM represented results with high quality, and they both had similar cumulative-variation-representing trends for nrSSM and rSSM, which means the high reliability of rSSM. The association between SSMs and kinematics during the daily activities can be found in the future study.

## Figures and Tables

**Figure 1:** Overview of the process for the statistical model generation. (a) A set of training CT images. (b) Simulated and meshed 3D resource models. (c) The template 3D model. (d) The resource models register and alignment to the template model. (e) The distance map between the mean model, −2SD model, and +2SD model after PCA.

**Figure 2:** Region definition with Gaussian curvature analysis (a). Red area represents positive, blue area represents negative. Definition of anatomical terms of location in the view of frontal plane (b).

**Figure 3:** Comparison of cumulative variation percentages of nonregion-based SSM and region-based SSM.

**Figure 4:** Morphological variations in the first four principal components in the first metacarpal bone (nrSSM). Row (a) represents the distance map of the mean model and −2SD model. Row (b) represents the distance map of the mean model and +2SD model. Row (c) represents the distance map of the −2SD model and the +2SD model.

**Figure 5:** Principal components of the first metacarpal bone with nrSSM from −2SD model to +2SD model: (a) represents the first principal component; (b) represents the second principal component; (c) represents the third principal component; (d) represents the fourth principal component.

**Figure 6:** Gaussian curvature value between nonregion-based SSM and region-based SSM.

## Data Availability

The data that support the findings of this study are available from the corresponding author upon reasonable request.
